# Combined Effect of Smoking and Fatty Liver Disease on the Progression of Type 2 Diabetes: Insights from a Population-Based Cohort Study

**DOI:** 10.1155/2022/1776875

**Published:** 2022-07-09

**Authors:** Tingting Zhang, Donghe Zhang, Jing Zeng, Yan Yang, Yi Fang, Xuan Wang

**Affiliations:** ^1^Department of Endocrinology, The Fifth Medical Center of Chinese PLA Hospital, Beijing, China; ^2^Department of Day Clinic, The Fifth Medical Center of Chinese PLA Hospital, Beijing, China

## Abstract

**Objectives:**

Fatty liver disease (FLD) is strongly linked to the occurrence of type 2 diabetes mellitus (T2DM). Insulin resistance (IR) is linked to smoking. Our study's purpose was to see how smoking and fatty liver accompanied affected the development of T2DM in the past.

**Materials and Methods:**

We collected data from 15,464 Japanese adults aged 18 to 79 years who took part in the NAGALA research, and our team utilized a Cox proportion risk model to look at the combination effect of FLD and smoking status on the incidence of T2DM. Participants were separated into three categories: nonsmokers, ex-smokers, and current smokers. An abdominal ultrasound was used to diagnose FLD.

**Results:**

384 subjects had T2DM after a median follow-up of 5.4 years. In comparison to the other groups, current FLD smokers had a greater chance of developing T2DM. Ex-smokers and present FLD smokers, on the other hand, had no significant difference in their likelihood of acquiring T2DM. When compared to ex-smokers and nonsmokers without FLD, current smokers with FLD had a considerably greater chance of acquiring T2DM. Furthermore, the risk of T2DM among nonsmokers, ex-smokers with FLD, and current smokers without FLD was not statistically significant.

**Conclusions:**

In order to prevent the progression of T2DM, we should recognize that smoking status may vary in FLD.

## 1. Introduction

As one of the most rapidly growing chronic diseases nowadays, early intervention for diabetes is of great interest. The International Diabetes Federation reports that in 2019, the global prevalence of diabetes is 9.3% among adults aged 20-79 years (an astonishing 463 million people), and this number is anticipated to attain 700 million by 2045 [1]. Individuals, society, and the nation all bear a significant financial burden due to type 2 diabetes mellitus (T2DM) and its sequelae. Unhealthy eating habits, obesity, and a sedentary life style are all key risk factors for type 2 diabetes [2, 3]. Therefore, it is important to prevent and treat T2DM. Fatty liver disease (FLD), is tightly related to IR in the body. Currently, it is considered one of the main reasons of ectopical fat cumulation [4, 5] and has been reported as a vital risky factor for the developmental process of T2DM [5].

As a major issue of social and human health, smoking itself now affects about 1.1 billion people worldwide [6]. Based on four main aspects of pathological mechanisms, increased abdomen fat cumulation, elevated sympathetic activity, chronic pancreatic cell inflammation, and straight toxic impairment to pancreas cells, smoker develops abnormal glucose metabolism and even promotes the development of diabetes [7, 8]. In patients who were diagnosed with diabetes, studies also have found that smoking causes inflammation and vascular endothelial dysfunction, which in turn increases the risks of micro blood vessel and major vessel illnesses in diabetic's sufferers [7, 9]. Cotinine-validated current smoking and self-reported current smoking have both been associated to nonalcoholic fatty liver disease (NAFLD) [10]. As a result, depending on background variables like FLD, the effect of smoking status on T2DM may differ. However, no prior research has looked at the combined impact of FLD and smoking status on the development of T2DM.

The influence of smoking status on the incidence of incident T2DM in people with and without FLD was investigated in the present study. The findings of this study could help doctors better understand how to counsel people about quitting smoking based on their unique circumstances, such as the presence of FLD.

The structure of this article is organized as follows. The materials and methods is presented in Section 2. The statistical analysis is explained in Section 3. The experimental results is presented in Section 4.  Section 5 consists of the discussion section. Finally, Section 6 summarizes the paper's main points.

## 2. Materials and Methods

### 2.1. Data Source

Our team acquired data from the publicly available “DRYAD” database (https://datadryad.org/). Data can be obtained from the following article: ectopic fat obesity presents the greatest risk for incident T2DM: a population-based longitudinal study [5] (data set: 10.5061/dryad.8q0p192).

### 2.2. Study Design and Participants

This research was on the foundation of the accessible data from the NAGALA study. From 2004 to 2015, it was a longitudinal research at Murakami Memorial Hospital's Medical Health Checkup Center (Gifu, Japan). The NAGALA research was discussed in depth in the original article. In total, 20,944 individuals were recruited for this study between 2004 and 2015, and all participated in a physical examination program and completed at least two exams.

Finally, exclusion criteria were used to select 15,464 individuals for data analysis. (1) People who were already on medication at the time of the baseline detection (*n* = 2321), (2) sufferers with abnormal glucose metabolism (T2DM *n* = 323 or impaired fasting glucose (IFG) *n* = 808), (3) people who drink heavily (*n* = 739), (4) patients with a diagnosis of chronic viral hepatitis (like hepatitis B or hepatitis C (*n* = 416)), (5) patients with missing covariate data, such as height, exercise, alcohol intake, or abdomen ultrasound (*n* = 863), and (6) patients with inaccurate data on waist circumference (WC) (*n* = 2). The investigation was done by Okamura et al. [5]. According to their description, the study was accepted by Murakami Memorial Hospital's ethics committee, and each participant gave their informed permission.

### 2.3. Measurements and Data Collection

All participants completed a standardized self-administered questionnaire to acquire medical information and life style variables, such as alcohol use, smoking status, and physical activity. Experienced nurses performed anthropometric measurements of participants such as weight, height, WC, and blood pressure. Body mass index (BMI) was computed via normal formula (weight/height squared (kg/m^2^). Fasting blood specimens were harvested and completed for measurements and analyses of biochemical indicators and other relevant indicators. These include total cholesterol, triglycerides, LDL-C, HDL-C, fasting blood glucose (FPG), and glycated hemoglobin (HbA1c).

### 2.4. Definition of FLD

Abdominal ultrasound was performed by a trained technician, and then, the gastroenterologist examined the ultrasound images without reference to other personal data of the subject. The diagnosis of FLD on ultrasound images is based on four criteria: vascular blurring, deep attenuation, liver and kidney sonography, and liver brightness [11].

### 2.5. Definition of T2DM

The diagnosis of T2DM in this study was on the foundation of ≥1 standards below that have been validated: FBG ≥ 7.0 mmol/L, HbA1c ≥ 6.5%, self-reported diabetic disease, or already treated for diabetes treatment [12].

Information on the smoking history of the study population was clarified by chart review and direct interviews with patients. The included study population was informed by a study information letter and then interviewed by telephone. From this interview and medical records, the study population was further divided into “nonsmokers” or “ex-smokers” and “current smokers.”

## 3. Statistical Analysis

All analysis was completed via R Statistical Software (http://www.r.project.org), and *P* < 0.05 had significance on statistics. In addition, continuous variates are presented as average ± SD, and categorical variates are presented as percentages (%).

Based on the presence of FLD and current smoking status, the participants were divided into six groups in our study and compared the differences between groups. The Kaplan-Meier technique was also utilized to provide a graphic representation of time to incident T2DM throughout follow-up, as well as the log-rank test to determine the importance of diversities between the six groups. Multivariable Cox regressive models were used to determine hazard ratios (HRs) and 95 percent confidence intervals (95 percent CI) for incident T2DM due to the presence of censored cases and the follow-up time being inconsistent. Models were provided that were both nonadjusted and multivariate adjusted. Confounding factors were defined as variables that altered the original regressive coefficients by more than 10%. Gender, age, BMI, alcohol consumption, fatty liver, SBP, triglycerides, HDL-C, FPG, and HbA1c were all adjusted in this study. Cox regression was used to test for trend by using the median value of six groups as categorical variables in the models. The stratified Cox regressive models were utilized to perform the subgroup analysis.

## 4. Results

### 4.1. Baseline Features of Participants

At a median follow-up of 5.4 years, 373 of the 15,464 subjects had T2DM. The average age of the entire participants was 43.71 ± 8.90 years, and 54.5% of the study population was male. All baseline information is shown in Table 1.

The proportions of nonsmoker, ex-smoker, and current smoker were 58.4% (9031), 19.1% (2952), and 22.5% (3481), respectively. We categorized six groups based on FLD status (with/without) and current smoking status, as well as the differences in baseline features between the six groups. The proportions (number) of nonsmoker, ex-smoker, and current smoker without FLD were 61.3% (7805), 17.5% (2226), and 21.2% (2692), respectively, and that of nonsmoker, ex-smoker, and current smoker with FLD were 44.7% (1226), 26.5% (726), and 28.8% (789), respectively. Patients with FLD were much heavier than those without the disease. Furthermore, in patients with FLD, WC was significantly higher than in patients without FLD. Nonsmokers, ex-smokers, and current smokers had higher fasting glucose levels and lower HbA1C levels (Table 1).

At a median follow-up of 5.4 years, 373 participants had T2DM. The cumulative incidence of 4000-day T2DM was 11.9%, 6.9%, and 6.4% in nonsmokers, ex-smokers, and current smokers without FLD, respectively (Figure 1). Compared with nonsmoker, ex-smoker displayed a remarkable risk for incident T2DM (HR 1.66, 95% CI 1.26 to 2.18, *P* < 0.001), and current smoker displayed a remarkable risk as well (HR 2.58, 95% CI 2.06 to 3.24, *P* < 0.001). FLD displayed a remarkable risk as well (HR 7.02, 95% CI 5.7 to 8.63, *P* < 0.001) (Table 2).

To examine the six groups' risk of developing T2DM, we employed Cox proportion risk models (univariable and multivariable Cox proportion risk models). The effect sizes (HR) and 95% CI intervals are listed in Table 3. Current smokers without FLD had a significantly higher risk of incident T2DM in gender- and age-adjusted Cox-hazard regression analysis (HR, 2.16; 95% CI, 1.45 to 3.22); in the fully adjusted model, Cox-hazard regression analysis, current smoker without FLD significantly increased risk for incident T2DM (HR, 1.78; 95% CI, 1.18 to 2.68) (Table 3). In gender- and age-adjusted Cox-hazard regression analysis, nonsmoker with FLD significantly increased risk for incident T2DM (HR, 7.44; 95% CI, 5.29 to 10.52); in the fully adjusted model, Cox-hazard regressive analyses, nonsmoker with FLD significantly increased risk for incident T2DM (HR, 2.02; 95% CI, 1.38 to 2.95) (Table 3). In gender- and age-adjusted Cox-hazard regressive analyses, current smoker with FLD remarkably elevated risk for incident T2DM (HR, 13.39; 95% CI, 9.19 to 19.5). In the fully adjusted model, Cox-hazard regressive analyses, current smoker with FLD significantly increased risk for incident T2DM (HR, 3.63; 95% CI, 2.41 to 5.48) (Table 3).

Figure 2 depicts the findings of HRs for each of the six groups on incident T2DM. Nonsmokers without FLD and ex-smokers without FLD had a reduced incidence of incident T2DM than the other categories. The nonsmoker group with FLD and the ex-smoker group with FLD, on the other hand, had a substantially greater risk of incident T2DM than the nonsmoker group without FLD and the ex-smoker group without FLD, respectively. Current smokers with FLD exhibited a considerably elevated risk when compared to the other groups. Current smokers with no FLD had a remarkably elevated risk of having T2DM than ex-smokers without FLD and nonsmokers with no FLD (vs. none HR 1.78, 95 percent CI 1.18 to 2.68, *P* = 0.006; vs. ex-smoker, HR 1.75, 95 percent CI 1.1 to 2.79, p = 0.018), but no evident diversity existed in the risk for developing T2DM between nonsmoker and ex-smoker with FLD (vs. HR 0.88, 95% CI 0.6 to 1.28, *P* = 0.495).

## 5. Discussion

In a cohort of 15464 Japanese people who were followed for a mean of 5.4 years, we looked at the risk of incident T2DM in relation to both the existence of FLD and the status of smoking. Many prior cross-section researches and longitudinal researchers have found that smoking is a risky factor for T2DM, with the great risk being about as 30% to 40% among current smokers vs. nonsmokers [7–9, 13]. We discovered that our sample with FLD had a greater rate of current smoking (28.8%) than those without FLD (21.2%). This indicates that primary and/or secondary preventative smoking cessation recommendations are not being followed to their full potential in this high-risk cohort. Meanwhile, we discovered that never smokers and ex-smokers without FLD were less likely to develop incident T2DM than never smokers and ex-smokers with FLD; but nonsmokers and ex-smokers with FLD had a greater risk of having incident T2DM than never smokers and ex-smokers without FLD. On the other hand, the risk of current smoker even with no FLD was greater, compared with that nonsmoker and ex-smoker with no FLD. In addition, our team has unveiled that the risk of incident T2DM in current smokers with FLD was the greatest among the six groups.

Many researchers have found that self-reported previous smoking does not elevate the risk of developing diabetes. Moreover, there are contradictory views as to whether previous smoking is related to an elevated risk of having diabetes [14–16]. The current study suggests that in the early phases of smoking quitting, accompanied by weight gain, particularly abdominal fat, patients may develop IGT, insulin resistance, and even diabetes. However, as the length of smoking cessation extended, it was discovered that stopping smoking was closely linked to a reduction in the risk of diabetes illness in this group [14]. As a result of the findings of this study, the function of smoking in IR, glycemic control, and diabetic development may be reversible. Through our study, we found no remarkable diversity between the prevalence of diabetes in the ex-smoker and never smoker groups for the population without FLD, suggesting the importance of timely smoking cessation in the absence of fatty liver to delay the onset of diabetes. Compared to the current smoking group, the ex-smoking group focused on adjusting poor lifestyle and improving various metabolic syndrome-related factors, like controlling blood pressure and lipid and glucose (GLU) levels, which may have played a balancing role in the relationship between smoking and diabetes prevalence. Given the persistently high prevalence of smoking and our report above, assessment of tobacco use and counseling or treatment to help quit smoking should be considered necessary for the development of T2DM, as recommended by the guidelines.

One of the greatest strengths of our study, it is a longitudinal study based on a relatively large Asian population. The combined effect of smoking status and fatty liver on T2DM was focused on, which is an important clinical guideline for preventing the development of diabetes from a lifestyle perspective. In addition, the same standardized diagnostic criteria were used for the diagnoses of fatty liver in the study, and a standardized questionnaire for life style factors was used.

However, there are certain faults in this paper. An abdominal ultrasound was used to confirm the diagnosis of FLD. Ultrasound, unlike liver biopsies, may not be accurate. Second, because our team failed to conduct an oral GLU tolerance assay at the time of diabetes diagnosis, the occurrence of T2DM may not be adequately estimated. Third, we did not record the amount of smoking and duration of smoking in self-reported current smokers (smoking/day). Fourth, the ability to detect the effects of diverse degrees of physical activities on the body's GLU metabolic homoeostasis and ectopical adiposity is insufficient. In the future, if we can adequately assess the intensities and frequencies of exercises, analyses with more accuracy can be performed. Fifth, we could not assess the incidence of passive smoking on diabetes in this study because passive smoking was not documented and we could not assess the incidence of passive smoking in this study. Finally, we did not have detailed data on the types of drugs. If our team acquired those information, a subanalysis of the excluded patients might offer novel enlightenment.

## 6. Conclusion

Holistically, among the six groups, current FLD smokers had the greatest risk of developing T2DM. In addition, never smoking was related to a lower risk of T2DM in sufferers without FLD, but not in sufferers with FLD. Ex-smokers had a reduced incidence of T2DM than current smokers in patients with FLD. Clinicians must be worried about the presence of FLD and the patient's smoking status in order to prevent the development of T2DM and should advise smoking cessation.

## Figures and Tables

**Figure 1:** The Kaplan-Meier analysis of incident type 2 diabetes in the NAGALA study, 2004–2015.

**Figure 2:** HRs and 95% CIs for incident type 2 diabetes. The numbers below each group indicate the number of participants who developed type 2 diabetes/participants classified in each group (percentage). The HRs and 95% CIs were calculated adjusting for sex, age, body mass index, waist circumference, exercise, fasting plasma glucose, hemoglobin A1c, SBP, DBP, total cholesterol, triglycerides, HDL cholesterol, and alanine transaminase at baseline. FL: fatty liver; non-: none.

**Table 1:** The Characteristic of participants in the NAGALA study, 2004–2015.

	Total	Nonsmoker	Ex-smoker	Current smoker
FLD− (*n*)	12723	7805	2226	2692
Sex, *n* (%)				
Women	6548 (51.5)	5709 (73.1)	416 (18.7)	423 (15.7)
Age (year)	43.5 ± 9.0	42.9 ± 8.7	45.2 ± 9.7	43.6 ± 9.0
Body weight (kg)	72.3 ± 11.2	70.5 ± 12.0	72.8 ± 9.5	74.7 ± 11.1
Body mass index (kg/m^2^)	21.4 ± 2.6	21.0 ± 2.6	22.1 ± 2.4	21.9 ± 2.7
Waist circumference (cm)	74.4 ± 8.0	72.6 ± 7.7	77.6 ± 7.3	77.0 ± 7.7
SBP (mm Hg)	112.5 ± 14.2	111.0 ± 14.1	116.4 ± 14.2	113.8 ± 14.0
DBP (mm Hg)	70.2 ± 10.0	68.9 ± 9.8	73.2 ± 10.0	71.3 ± 9.9
Exercise type, *n* (%)				
Irregular exercise	10415 (81.9)	6413 (82.2)	1699 (76.3)	2303 (85.5)
Regular exercise	2308 (18.1)	1392 (17.8)	527 (23.7)	389 (14.5)
HDL cholesterol (mmol/L)	1.5 ± 0.4	1.6 ± 0.4	1.5 ± 0.4	1.3 ± 0.4
Total cholesterol (mmol/L)	5.1 ± 0.8	5.1 ± 0.9	5.1 ± 0.8	5.0 ± 0.8
Triglycerides (mmol/L)	0.8 ± 0.5	0.7 ± 0.4	0.9 ± 0.6	1.0 ± 0.7
Fasting plasma glucose (mmol/L)	5.1 ± 0.4	5.0 ± 0.4	5.2 ± 0.4	5.2 ± 0.4
HbA1C (%)	5.1 ± 0.3	5.2 ± 0.3	5.1 ± 0.3	5.1 ± 0.3
Alcohol consume type, *n* (%)				
None or minimal alcohol consumer	9717 (76.4)	6838 (87.6)	1332 (59.8)	1547 (57.5)
Light alcohol consumer	1472 (11.6)	599 (7.7)	411 (18.5)	462 (17.2)
Moderate alcohol consumer	1110 (8.7)	295 (3.8)	347 (15.6)	468 (17.4)
Heavy alcohol consumer	424 (3.3)	73 (0.9)	136 (6.1)	215 (8)
ALT (IU/L)	15.0 (12.0, 20.0)	14.0 (11.0, 19.0)	17.0 (14.0, 22.0)	17.0 (13.0, 23.0)
AST (IU/L)	17.0 (14.0, 20.0)	16.0 (14.0, 20.0)	18.0 (14.0, 22.0)	17.0 (14.0, 20.0)
GGT (IU/L)	14.0 (11.0, 20.0)	13.0 (10.0, 16.0)	17.0 (13.0, 24.0)	17.0 (13.0, 24.0)
FLD+ (*n*)	2741	1226	726	789
Sex, *n* (%)				
Women	486 (17.7)	430 (35.1)	25 (3.4)	31 (3.9)
Age (year)	44.8 ± 8.3	44.4 ± 8.4	46.4 ± 8.7	44.0 ± 7.6
Body weight	72.3 ± 11.2	70.5 ± 12.0	72.8 ± 9.5	74.7 ± 11.1
Body mass index (kg/m^2^)	25.5 ± 3.1	25.5 ± 3.3	25.2 ± 2.7	25.7 ± 3.2
Waist circumference (cm)	86.1 ± 7.7	85.3 ± 8.2	86.2 ± 6.6	87.2 ± 7.8
SBP (mm Hg)	123.8 ± 14.8	124.5 ± 15.2	124.6 ± 14.4	121.9 ± 14.4
DBP (mm Hg)	78.1 ± 10.2	78.2 ± 10.3	79.2 ± 10.1	77.0 ± 10.0
Exercise type, *n* (%)				
Irregular exercise	2340 (85.4)	1046 (85.3)	605 (83.3)	689 (87.3)
Regular exercise	401 (14.6)	180 (14.7)	121 (16.7)	100 (12.7)
HDL cholesterol (mmol/L)	1.2 ± 0.3	1.3 ± 0.3	1.2 ± 0.3	1.1 ± 0.3
Total cholesterol (mmol/L)	5.4 ± 0.9	5.4 ± 0.9	5.4 ± 0.8	5.5 ± 0.9
Triglycerides (mmol/L)	1.5 ± 0.8	1.3 ± 0.8	1.5 ± 0.9	1.6 ± 0.9
Fasting plasma glucose (mmol/L)	5.4 ± 0.4	5.4 ± 0.4	5.4 ± 0.4	5.4 ± 0.3
HbA1C (%)	5.3 ± 0.3	5.3 ± 0.3	5.3 ± 0.3	5.3 ± 0.3
Alcohol consume type, *n* (%)				
None or minimal alcohol consumer	2088 (76.2)	1069 (87.2)	480 (66.1)	539 (68.3)
Light alcohol consumer	286 (10.4)	82 (6.7)	104 (14.3)	100 (12.7)
Moderate alcohol consumer	250 (9.1)	55 (4.5)	101 (13.9)	94 (11.9)
Heavy alcohol consumer	117 (4.3)	20 (1.6)	41 (5.6)	56 (7.1)
ALT (IU/L)	27.0 (20.0, 39.0)	25.0 (19.0, 36.8)	28.5 (22.0, 41.0)	28.0 (21.0, 40.0)
AST (IU/L)	21.0 (17.0, 26.0)	20.0 (17.0, 26.0)	21.0 (17.0, 27.0)	20.0 (16.0, 25.0)
GGT (IU/L)	23.0 (17.0, 35.0)	21.0 (15.0, 30.8)	25.0 (19.0, 37.0)	25.0 (19.0, 38.0)

Data are expressed as the number (%) of subjects or mean (SD). ALT: alanine transaminase; AST: aspartate transaminase; DBP: diastolic blood pressure; FLD: fatty liver disease; GGT: gamma-glutamyl transferase; HDL: high-density lipoprotein; SBP: systolic blood pressure.

**Table 2:** Univariate analysis for incident type 2 diabetes in the NAGALA study, 2004–2015.

	HR (95% CI)	*P* (Wald's test)	*P* (LR-test)
Sex: men vs. women	2.52 (1.98, 3.21)	< 0.001	< 0.001
Age (year)	1.06 (1.04, 1.07)	< 0.001	< 0.001
Fatty liver: yes vs. no	7.02 (5.70, 8.63)	< 0.001	< 0.001
Body mass index (kg/m^2^)	1.24 (1.22, 1.27)	< 0.001	< 0.001
Waist circumference (cm)	1.09 (1.08, 1.10)	< 0.001	< 0.001
ALT (mmol/L)	1.01(1.01, 1.01)	< 0.001	< 0.001
AST (mmol/L)	1.01 (1.01, 1.01)	< 0.001	< 0.001
GGT (mmol/L)	1.01 (1.01, 1.01)	< 0.001	< 0.001
HDL-C (mmol/L)	0.15 (0.11, 0.20)	< 0.001	< 0.001
TC (mmol/L)	1.49 (1.34, 1.66)	< 0.001	< 0.001
TG (mmol/L)	1.80 (1.68, 1.92)	< 0.001	< 0.001
HBA1C (%)	54.30 (39.51, 74.62)	< 0.001	< 0.001
Exercise : regular vs. irregular	0.76 (0.56, 1.02)	0.064	0.056
Alcohol consumption (%) ref. = 1			0.001
Light	0.90 (0.65, 1.26)	0.551	
Moderate	1.15 (0.82, 1.62)	0.424	
Heavy	2.24 (1.54, 3.27)	< 0.001	
Smoking status (%) ref. = 1			< 0.001
Ex-smoker	1.66 (1.26, 2.18)	< 0.001	
Current-smoker	2.58 (2.06, 3.24)	< 0.001	
FBG (mmol/L)	25.38 (18.71, 34.42)	< 0.001	< 0.001
SBP (mm Hg)	1.03 (1.03, 1.04)	< 0.001	< 0.001
DBP (mm Hg)	1.05 (1.04, 1.06)	< 0.001	< 0.001

BMI: body mass index; WC: waist circumference; HDL-C: high-density lipoprotein cholesterol; TC: total cholesterol; TG: triglyceride; FPG: fasting plasma glucose; SBP: systolic blood pressure; DBP: diastolic blood pressure; T2DM: type 2 diabetes mellitus; CI: confidence interval; HR: hazard ratio.

**Table 3:** Association between FL with smoking statues and incident type 2 diabetes in the NAGALA study, 2004–2015.

Exposure	Nonadjusted		Adjust I		Adjust II	
	HR (95% CI)	*P* value	HR (95% CI)	*P* value	HR (95% CI)	*P* value
Smoking status						
FL−/none	1 (reference		1 (ref)		1 (ref)	
FL−/ex	1.50 (0.96, 2.35)	0.074	1.23 (0.76, 2)	0.401	1.01 (0.62, 1.66)	0.956
FL−/current	2.37 (1.66, 3.37)	<0.001	2.16 (1.45, 3.22)	<0.001	1.78 (1.18, 2.68)	0.006
FL+/none	7.94 (5.73, 11.02)	<0.001	7.44 (5.26, 10.52)	<0.001	2.02 (1.38, 2.95)	<0.001
FL+/ex	7.83 (5.42, 11.31)	<0.001	6.21 (4.05, 9.51)	<0.001	1.77 (1.13, 2.77)	0.013
FL+/current	14.30 (10.44, 19.6)	<0.001	13.39 (9.19, 19.5)	<0.001	3.63 (2.41, 5.48)	<0.001
*P* for trend	<0.001		<0.001		<0.001	

Notes: data presented are HR (95% CI); Adjust I model adjust for age and gender; Adjust II model adjust for Adjust I+BMI, SBP, DBP, WC, ALT, AST, GGT, and HDL-C+TC+TG+HBA1C+FBG. Abbreviation: FL: fatty liver.

## Data Availability

The data used to support the findings of this study are available from the corresponding author upon request.
